# Computed Tomography Angiography under Deep Learning in the Treatment of Atherosclerosis with Rapamycin

**DOI:** 10.1155/2021/4543702

**Published:** 2021-07-22

**Authors:** Fuguang Ji, Shuai Zhou, Zhangshuan Bi

**Affiliations:** ^1^Intensive Care Unit, People's Hospital of Zhongmou, Zhengzhou 451450, Henan, China; ^2^Department of Cardiology, The First Affiliated Hospital of Zhengzhou University, Zhengzhou 450052, Henan, China

## Abstract

The clinical characteristics and vascular computed tomography (CT) imaging characteristics of patients were explored so as to assist clinicians in diagnosing patients with atherosclerosis. 316 patients with atherosclerosis who were hospitalized for emergency treatment were treated with rapamycin (RAPA) in the hospital. A group of manually delineated left ventricular myocardia (LVM) on the patient's coronary computed tomography angiography (CCTA) were selected as the region of interest for imaging features extracted. The CCTA images of 80% of patients were randomly selected for training, and those of 20% of patients were used for verification. The correlation matrix method was used to remove redundant image omics features under different correlation thresholds. In the validation set, CCTA diagnostic parameters were about 40 times higher than the manually segmented data. The average dice similarity coefficient was 91.6%. The proposed method also produced a very small centroid distance (mean 1.058 mm, standard deviation 1.245 mm) and volume difference (mean 1.640), with a segmentation time of about 1.45 ± 0.51 s, compared to about 744.8 ± 117.49 s for physician manual segmentation. Therefore, the deep learning model effectively segmented the atherosclerotic lesion area, measured and assisted the diagnosis of future atherosclerosis clinical cases, improved medical efficiency, and accurately identified the patient's lesion area. It had great application potential in helping diagnosis and curative effect analysis of atherosclerosis.

## 1. Introduction

The coronary atherosclerotic heart disease (CAHD) is a common cardiovascular disease endangering human physical and mental health in China. It is the most common type of organ disease caused by atherosclerosis, and the acute myocardial infarction (AMI) is the most serious type of coronary heart disease [1, 2]. In recent years, with the continuous development of China's economy and the continuous rise of the people's happiness index, the incidence of atherosclerosis in China has also increased year by year, with 45–55 deaths per 100,000 people from atherosclerosis. Besides, people who get sick are getting younger and younger, making the occurrence and prognosis of AMI a central issue in current research [3].

Rapamycin (RAPA) is the first known mammalian target of rapamycin (mTOR) pathway inhibitor, and the molecular formula is C_51_H_79_NO_13_. As a traditional macrolide antibiotic, RAPA was first isolated from the fungus *Streptomyces hygroscopicus* and used as an antifungal drug in the 1970s. It was certified by the U.S. Food and Drug Administration in 1999 to resist acute immune rejection of organ transplant patients [1]. In recent years, the antitumor activity and antiaging function of RAPA and its analogues have been gradually discovered; they also have certain effects on diabetes and cardiovascular diseases (CVD) and so forth and have been gradually applied in relevant clinical treatment [4].

The imaging examination plays an important role in assessing whether patients with coronary heart disease are accompanied by myocardial ischemia [5]. However, ultrasound examination has strong subjective dependence, which is related to the experience of the operator. Its current application value in diagnosing myocardial ischemia is limited. Coronary computed tomography angiography (CCTA) can clearly show the structure of the heart and the condition of the coronary arteries [6]. Clinicians can assess the degree of stenosis of the coronary arteries and the characteristics of stenosis plaques, and then they can stratify patients for risk. However, the radiology department or clinician cannot directly identify whether the patient is accompanied by myocardial ischemia on the resting CCTA. CCTA combined with stress perfusion examination can visually display whether the myocardium has perfusion defects and can identify myocardial ischemia. However, compared with resting state CCTA, stress perfusion examination will increase the radiation dose, and the use of stress drugs will increase the risk of patient examination, and some patients cannot tolerate it [7]. Therefore, if advanced image analysis methods, such as artificial intelligence (AI) technologies, can be used to identify myocardial ischemia on the CCTA in the conventional resting state, the various follow-up invasive examinations can be reduced, which has important clinical significance.

AI is a branch of the field of computer science, which aims to imitate human thinking process, learning ability, and knowledge storage as much as possible [8]. Some research limitations based on traditional methods have gradually become prominent with the advent of the “big data” era. With the development of computer hardware and software, the application research of AI in the medical field has become a hot topic [9]. At present, the research results of AI in the medical field continue to emerge, and it has applications in disease screening, diagnosis, choice of treatment methods, and patient prognosis judgments. At present, many studies showed that some diagnostic or predictive models based on AI methods were better than those based on traditional methods. For example, Esteva et al. [10, 11] established a machine learning-based model to predict the 5-year all-cause mortality of patients with suspected coronary heart disease. This model evaluated 25 clinical features and 44 CCTA-based features. This model based on machine learning had better predictive performance than the Framingham risk assessment model established by traditional statistical methods. However, the above-mentioned work required the clinician to manually outline the contour of the myocardium on the corresponding image, which was undoubtedly a heavy and laborious work [12]. At present, studies showed that some deep learning-based methods can quickly, efficiently, and automatically outline the structure of interest, which not only greatly reduced the workload of clinicians, but also avoided subjective differences between different doctors to a certain extent [13].

Therefore, the research aimed to study the use of imaging omics methods combined with machine learning methods to analyze LVM characteristics. As a reference, the fractional flow reserve (FFR) of invasive coronary artery was compared with the hemodynamically significant stenosis judged by CCTA and invasive coronary angiography (ICA) to evaluate the effectiveness of different methods in diagnosing atherosclerosis. In addition, through the deep learning method and with the contour of the left ventricle myocardium manually drawn by the clinician as a reference, a deep learning model that can accurately and automatically outline the left ventricle was constructed to reduce the workload of the clinician.

## 2. Methods

### 2.1. Research Object

316 patients with CAHD who underwent emergency treatment for the first time within 12 hours of onset of hospitalization were selected in the research from May 2017 to March 2021. There were 221 males and 95 females, aged 60.66 ± 12.19 years. The CAHD patients met the 2014 American College of Cardiology/American Heart Association (ACC/AHA) AMI diagnostic criteria.

Inclusion criteria were as follows: a) patients who met the diagnostic criteria of AMI and received emergency treatment within twelve hours; b) patients with complete case data and complete follow-up on time.

Exclusion criteria were as follows: (a) patients with a history of myocardial infarction or coronary revascularization; (b) patients with previous arrhythmia such as persistent atrial fibrillation; (c) patients with hematological diseases, malignant tumors, autoimmune diseases, infections, or inflammatory diseases; (d) patients with severe heart, liver, and kidney dysfunction; (e) patients with recent major trauma and major surgery; (f) patients with incomplete clinical data.

A total of 316 patients with coronary atherosclerosis met the above inclusion criteria and exclusion criteria in the research. The research had been approved by the medical ethics committee of hospital, and the family members of the patients included in the research had signed an informed consent form.

### 2.2. Data Acquisition and Image Analysis

#### 2.2.1. CCTA Data Collection

The CCTA data was collected for all patients using 64 rows, and CCTA images were collected by scanning machines from four different CT manufacturers (Siemens, Somatom Flash, Definition Flash, Somatom Definition FlashAS+, Force; GE Discovery CT 750 HD, Light Speed VCT; Toshiba, Aquilion One Vision; Philips BrillianceiCT 256). The patients took nitroglycerin sublingually to dilate the coronary arteries five minutes before the CCTA examination. For patients with a fast heart rate, they can consider taking oral p-blockers (25–75 mg) before the examination according to the doctor's recommendation. The CT scan range was determined according to location phase, which was from tracheal protrusion to lower edge of the heart. All patients received adaptive sequence acquisition triggered by prospective electrocardiogram.

#### 2.2.2. Image Analysis

The CCTA images of all patients were locally anonymized to remove sensitive information, then transmitted to the core laboratory, and imported into the Siemens postprocessing workstation for further analysis. The CCTA image quality was assessed by two experienced imaging doctors (with 3 years and 18 years of CCTA-related work experience, respectively). A 4-point method was used for evaluation: 1 = undiagnosable; 2 = acceptable; 3 = good; 4 = excellent. When there was a difference, the two radiologists reached a consensus through consultation. The cases with an image quality score of one were excluded.

### 2.3. Experiment Environment

#### 2.3.1. Construction of the Deep Learning Segmentation Model

Before the deep learning model was constructed, the contours of the left ventricular myocardium (LVM) of 100 patients were manually sketched as a reference for the deep learning method to learn from CCTA images. The deep learning model was composed of U-Net and deep attention, which mainly included two parts: training phase and segmentation phase. The flow chart of the research is shown in Figure 1. Before the training was started, the 3D-patches on the CCTA images and the corresponding hand-drawn myocardial contours were collected. A voxel window with a window size of 512 × 512 × 32 was used to slide on the *Z* axis of the image to extract 3D-patches. The data augmentation methods were used, such as flipping, rotating, and scaling, to increase the heterogeneity of the training set.  Figure 2 shows that the deep learning network was composed by an encoding path and a decoding path. The long-hop connection bypassed the feature extracted from the encoding path and was mapped to the decoding path.

#### 2.3.2. Deep Learning Model

After training, first the 3D-patches of the CCTA image were input into the trained model to obtain the probability map that each pixel on the CCTA image was the myocardial tissue, so as to obtain the myocardial segmentation result of the new patient. Then, these probability maps were merged into the entire image, and the final segmentation result of the LVM contour was obtained by gathering the myocardial probability maps and merging them on average. The fivefold cross-validation was used to verify the segmentation performance of the deep learning model. That is, the data of the above-mentioned patients were randomly classified into five equal parts, and four groups were selected for training, and the remaining group was used for verification. The dice similarity coefficient (DSC), mean surface distance (MSD), residual mean square distance (RMSD), center mass distance (CMD), and volume of difference (VOD) were used to evaluate the difference between LVM contour drawn by the model and that drawn manually by the doctor. The image segmentation accuracy was evaluated visually, and the segmentation time was recorded.

#### 2.3.3. Statistical Analysis

The data conforming to the normal distribution was represented by the mean ± standard deviation in the research, and the data not conforming to the normal distribution was represented by the median or percentage. The categorical variables were expressed in frequency and percentage. The commercial software (Med Calc; version 18.2.1) and SPSS 22.0 version were used for statistical analysis of data. The Kolmogorov–Smirnov test was used to determine whether the data fit a normal distribution. The *t*-test was used to compare the difference between LVM time by the automatic segmentation model and that drawn manually by the doctor. The bilateral *P* < 0.05 was considered statistically significant in the research.

### 2.4. Therapeutic Reagents and Methods

#### 2.4.1. Preparation of Therapeutic Reagent RAPA Nanoparticles (RAPA NP)

10 mg of RAPA and 20 mg of indomethacin (IND) were accurately weighed and added into 1 mL dimethyl sulfoxide (DMSO), which were fully suspended and dissolved with ultrasound. Then, 1 mL of DMSO suspension solution of 10 mg/mL PEI was added. After full and uniform mixing, the mixed solution was transferred into a dialysis bag (molecular weight was 3500 Da). The suspension of RAPA nanoparticles (PEI/IND/RAP) was obtained after dialyzed with ultrapure water for 24 hours. The suspensions containing different masses of small molecule shuttle-based drugs ursodeoxycholic acid (UDCA) were prepared in the same way.

#### 2.4.2. Treatment Method

300 mg aspirin and 180 mg ticagrelor/300 mg clopidogrel were given before treatment. RAPA was injected intravenously during treatment. Coronary angiography was performed via femoral artery or radial artery using standard techniques to assess coronary artery disease. Other treatments included angiotensin converting enzyme inhibitors (ACED) receptor blockers, diuretics, and nitrates, which can be used depending on the patient's own specific conditions.

### 2.5. Observation Index

The 0, 12, and 24 weeks were selected as the evaluation time points. The intima-media thickness (IMT) and plaque thickness (course integral) were detected at each evaluation point, and the patients in the treatment group were followed up to test the carotid artery intima-media thickness after three months to monitor the degree of treatment.

### 2.6. Statistical Method

The appropriate statistical analysis method was selected according to the nature of clinical trial data (measurement, classification, and grade data). The chi-square test or exact probability test was used for classification data, normality test and homogeneity test of variance were used for measurement data first, *t*-test was used for comparison of sample means for those who met the requirements, and paired *t*-test was used for the comparison of sample mean before and after treatment. The paired signed rank sum test was used to compare the samples that did not meet the conditions. The Wilcoxon rank sum test (correction) for sample comparisons or the Kruskal–Wallis test for multigroup comparisons were used for grade data. The repeated measure analysis of variance was used for quantitative primary outcome indexes at multiple observation time points. A two-sided test was used, with the baseline comparison test level *P*=0.05, the efficacy group comparison test level *P*=0.05, and the pairwise comparison between groups *P*=0.01670.

## 3. Results

### 3.1. Visual Assessment of the Results of the Deep Learning Model and the Doctor's Manual Segmentation

In the axial CCTA image, the comparison of the contour results of visual assessment method and the left ventricular muscle manually segmented by the doctor is shown in Figure 3. On the CCTA image, the contrast between the LVM and the surrounding tissues was not very different, while the segmentation effect of the proposed deep learning-based segmentation method was basically consistent with the contour of the myocardium manually segmented by the doctor.

### 3.2. Objective Parameters Evaluating the Results of the Deep Learning Model and Manual Segmentation by Doctors

In the data set of all patients, the LVM contour segmented by the proposed method was consistent with the myocardial contour drawn by doctors. The average DSC = 91.6%, and the standard deviation was 4.1%. The proposed method also produced very small CMD (average of 1.058 mm, standard deviation of 1.245 mm) and VOD (average of 1.640, standard deviation of 1.777), and the specific results are shown in Figure 4. The distance of HI was less than 10 mm, which meant that the pixels of the myocardium segmented by this method were very close to the pixels of the manually segmented myocardium, and LVM can be well positioned by this method.

In addition, the MSD and RMSD were both less than 2 mm, which indicated that the accuracy of the segmentation method was high. The differences of DSC and VOD between this method and manual segmentation of myocardium were evaluated at different levels of myocardium, and the results are shown in Figure 5.

### 3.3. The Time Required for Automatic Segmentation of Deep Learning Models and Manual Segmentation of LVM by Physicians

The time required for LVM by the automatic segmentation model and that of manual segmentation by the doctor were compared in the research. Through a randomized analysis of the time required for myocardial segmentation in 20 patients, it was found that LVM segmentation based on deep learning method required significantly short time. The deep learning method only needed an average of about 1.45 ± 0.51 seconds to complete segmentation, while the doctor's manual segmentation needed about 744.8 ± 117.49 seconds to complete segmentation (*P* < 0.001). The results showed that the efficiency and quality of automatic segmentation were much higher than those of manual segmentation by doctors.

### 3.4. Data Results after RAPA Treatment

#### 3.4.1. IMT Results

A paired *t*-test was performed in the control group and the treatment group to test the data before and after treatment. Wilcoxon signed rank test was used for the measurement data that did not meet the conditions before and after treatment. The Shapiro-Wilk normality test is shown in Figure 6. After inspection, the difference of the left carotid artery before and after IMT treatment in the treatment group showed that *P*=0.043, and the difference of the right carotid artery before and after IMT treatment showed that *P*=0.025. There were statistical differences before and after treatment, which proved that the use of a deep learning-based imaging system had a certain therapeutic effect in improving the thickness of carotid artery intima-media in patients with carotid atherosclerotic plaque.

#### 3.4.2. Carotid Artery Intima-Media Thickness Results

Before treatment, at the end of treatment, and during follow-up, the thickness of carotid medial artery was statistically analyzed and compared between groups, as shown in Figure 7. The IMT of left carotid artery was significantly different between the three groups at the end of treatment and 3 months of follow-up (*P*=0.025). At the end of treatment, there was a difference between the control group and the treatment group (*P*=0.011), while there was no statistical difference between the control group and the treatment group (*P*=0.618). After three months of follow-up, there was a difference between the control group and the treatment group (*P*=0.019), while there was no statistical difference between the control group and the treatment group (*P*=0.865). It was concluded that, in terms of the improvement of carotid artery thickness, the group using deep learning-based CT imaging characteristics analysis was superior to the control group with respect to the left carotid artery.

## 4. Discussion

How to accurately monitor the occurrence of adverse cardiac events in patients with atherosclerosis is always the core of cardiovascular disease research. The process of diagnosis and treatment of cardiovascular patients generates a large amount of data, including the patient's symptoms, laboratory test results, medical imaging data, and drug prescriptions. In general, clinicians judge the prognosis of patients based on their own models, their own experience, and the current condition of the patient. However, most prediction models were based on regression models and only used limited variables, which may not meet the requirements of accurate prediction [14]. The routine diagnosis and treatment of patients with CVD generated a large amount of data. At the same time, the amount of cardiovascular imaging data was also increasing. Clinically, doctors were unlikely to be familiar with various electronic medical record information including genetic data and cardiovascular imaging data and made full use of this information in clinical practice. This may lead to misdiagnosis due to insufficient information utilization. A recent study pointed out that about 40,000–80,000 people die every year because of diagnostic errors [15]. The autopsy studies found that diagnosis based on imaging data had an error rate of up to 20%. However, a fivefold cross-validation method was used to verify the segmentation effect of the LVM based on the proposed deep learning model. The subjective and objective methods were used to evaluate the contour difference between the proposed method of automatic segmentation of the LVM contour and the manual segmentation drawn by the doctor. It was verified that the proposed method could accurately segment the LVM tissue from CCTA images by analyzing six objective parameters, including DSC, HD, MSD, RMSD, C1VID, and VOD, and the proposed method significantly shortened the time needed to segment LVM from CCTA images. It reduced the time that would normally take about 12 minutes on average to about a second, which greatly reduced the workload of the doctor [16].

In the past, some scholars had achieved good results by establishing a deep learning-based method to automatically segment cardiac tissue of cardiac MRI images [17]. However, the contrast of myocardial tissue on CCTA images was not obvious compared with cardiac MR images, so there were few studies on the automatic segmentation of LVM on CCTA images. For the first time in the research, a neural learning network was used to integrate a deep-attention network to detect and segment LVM on CCTA images. After the model was trained, automatic LVM recognition and segmentation were performed on newly inputted CCTA images of patients. At present, some scholars have proposed to use different AI-based methods to segment the LVM on CCTA images. The imaging omics method used in this study can extract many quantitative and qualitative features from the region of interest on the image with high throughput. These imaging omics features can reflect the internal features of the organizational structure. Combined with machine learning methods, a lot of information was provided for the diagnosis of myocardial ischemia, which overcame the limitation of clinicians to analyze CCTA solely based on the naked eye. For example, Smyth et al. [18] used a multiscale convolutional neural network (CNN) to segment the LVM. The segmentation performance of CNN network on CCTA images of 20 patients was analyzed, and the average DSC was 0.910. Gertsen et al. [19] used a fully convolutional network to analyze the virtual single-energy CCTA data, and the best DSC value was 90.1 through CCTA image verification in 40 patients. The 3D fully convolutional neural network was used for CT brain tissue image segmentation, which can improve the accuracy of image analysis of atherosclerotic hard blood vessel function, and significantly improved the clearance rate of vascular plaque deposition and the recovery of carotid artery intima-media thickness after treatment. In this retrospective study, the feasibility of using imaging omics combined with machine learning method to analyze the characteristics of left ventricular myocardium on CCTA images to predict whether patients with coronary heart disease had myocardial ischemia was established and verified. Compared with the method that clinicians identify lesions based on CT images and determine myocardial ischemia based on the degree of coronary artery stenosis, the proposed method of image omics combined with machine learning had a better performance in predicting myocardial ischemia. The ability of the model to predict myocardial ischemia was relatively stable, and the accuracy was still high in the validation group. In addition, CCTA images generated by a number of hospitals and a variety of CT devices across the country were collected, and the model was randomly trained and verified, which reflected the universality and generalization of the model. To our knowledge, this was the first time that left ventricular myocardial features were analyzed using image omics to investigate whether patients with coronary heart disease had myocardial ischemia. Unlike the traditional clinical use of the degree of coronary artery stenosis as a standard to determine whether patients with CHD had myocardial ischemia, the characteristics of myocardium supplied by coronary arteries were analyzed to assess whether patients with CHD had myocardial ischemia, which also provided a new idea for future research.

## 5. Conclusion

The research showed that the CT angiography images were used during the treatment of atherosclerosis with rapamycin. Compared with the LVM contour manually drawn by the doctor on the CCTA image, the method proposed in the research had little difference with the LVM contour manually drawn by the doctor regardless of whether subjective or objective evaluation methods were used. The method significantly reduced the time required to segment LVM compared with traditional manual segmentation. However, there are still some shortcomings in this study. First, although patients with atherosclerosis were included in this study, CCTA images of only 100 patients were randomly and continuously selected for model training and validation. The results need to be further validated for the segmentation of myocardium on CCTA images collected by hospitals and CT scanning equipment in the future. Due to the different expertise and experience of imaging doctors, each doctor will have different contour labeling of the left ventricular myocardium, and such difference cannot be corrected by this deep learning algorithm. Second, there are only patients with suspected or confirmed coronary heart disease involved. The results of the myocardial segmentation model in patients with other diseases and at different stages of the disease need further study. Finally, the model is currently in the initial stage of establishment, and the extent to which it can reduce the workload of doctors in clinical practice is still unknown. Future research needs to be improved.

## Figures and Tables

**Figure 1:** Data analysis model.

**Figure 2:** Data gain model.

**Figure 3:** Manual segmentation (a) and deep learning segmentation (b).

**Figure 4:** The results of objective parameter evaluation of automatic and manual myocardial segmentation.

**Figure 5:** Evaluation of the parameter results of automatic and manual myocardial segmentation at different myocardial levels.

**Figure 6:** Comparison before and after IMT treatment.

**Figure 7:** The thickness of the left carotid artery intima-media at different time points in the two groups.

## Data Availability

No data were used to support this study.
